# Optimization Algorithm of Tourism Security Early Warning Information System Based on Long Short-Term Memory (LSTM)

This article has been retracted.

**DOI:** 10.1155/2021/9984003

**Published:** 2021-09-08

**Authors:** Lei Feng, Yukai Hao

**Affiliations:** ^1^School of Management, Wuhan University of Technology, Wuhan 400070, China; ^2^School of Economics and Management, Tibet University, Lhasa 850000, China

## Abstract

Tourism safety is the focus of the tourism industry. It is not only related to the safety of tourists' lives and property, but also related to social stability and sustainable development of the tourism industry. However, the security early warning of many scenic spots focuses on the response measures and remedial plans after the occurrence of security incidents, and the staff of many scenic spots have limited security awareness and information analysis ability, which is prone to lag in information release, and do not pay attention to the information of potential security problems. Therefore, this paper studies the optimization algorithm of the tourism security early warning information system based on the LSTM model and uses the recurrent neural network and LSTM to improve the processing and prediction ability of time-series data. The experimental results show that the number of three hidden layers in the tourism security early warning information system based on the LSTM model can reduce the training time of the model and improve the performance. Compared with the tourism safety early warning information system based on the BP neural network, it has better accuracy and stability, has better processing and prediction ability for time series data, and can monitor and analyze data scientifically in real-time and dynamically analyze data.

## 1. Introduction

Tourism has gradually become one of the important industries. As people no longer meet the basic needs of life, more and more people begin to pursue high-quality life. Tourism has gradually become one of the important industries. More and more people begin to pursue tourism life [1]. In addition, the tourism resources are constantly developed and utilized, and the tourism environment and content are constantly changing. In recent years, in addition to characteristic cultural city tourism, there are also natural and cultural tourism, marathon competition in natural tourism areas, etc. These emerging tourism projects not only attract more tourists but also improve the economic growth of the tourism industry [2, 3]. However, there are many unfortunate events that tourists encounter in the process of tourism, such as abrupt weather changes in marathon competitions in natural scenic spots, stampede on the Bund of Shanghai caused by too many tourists, tsunami, kidnapping of tourists, and constant theft in tourist areas, which have caused serious adverse effects on the tourism industry and restricted the sustainable development of the tourism industry [4, 5]. Therefore, tourism security has become a highly valued and concerned issue in various countries and regions, and tourism security early warning has become an inevitable trend of tourism development. With the development and application of intelligent information technology, many scenic spots will collect and release the safety information and early warning information of scenic spots through intelligent wearable products and corresponding apps based on big data, such as the information of dangerous areas of scenic spots and the number of visitors to scenic spots. Although the danger that some tourists will encounter in the scenic spots can be avoided to a certain extent, there are some problems in many scenic spots, such as untimely release of safety early warning information, low safety awareness of staff, and error in judgment of corresponding information. At the same time, the focus of many tourism safety measures, implementation plans, and methods in scenic spots is that after the occurrence of tourism safety events, the corresponding information release channel is narrow, and there is a lack of relevant knowledge reserve and mature and stable response plan in advance warning [6]. This shows that the development of tourism security early warning in the tourism industry can no longer meet the needs of the development of the tourism industry. Therefore, the tourism security early warning information system that the tourism industry needs to build can conduct accurate and scientific information analysis on the collected security information of relevant scenic spots in real-time and effectively, and output the information analysis results in time and improve the efficiency of safety early warning information in scenic spots.

This paper studies the optimization algorithm of the tourism security early warning information system based on the LSTM model. Compared with the traditional tourism security early warning methods, the artificial neural network has better fault tolerance and stronger robustness. It can quickly process data and find the corresponding optimal solution, and its nonlinear thinking can well deal with the relationship between many factors. Compared with the BP neural network, the LSTM model can better process temporal information and realize the purpose of real-time processing tourism safety early warning information. This paper is mainly divided into the following three parts. The first part introduces the development and related concepts of tourism security early warning information system and the development and application of the LSMT recurrent neural network. The second part constructs a tourism early warning information system based on the BP neural network and introduces the recursive neural network and LSTM to optimize the algorithm of the tourism early warning information system. In addition, the corresponding tourism security early warning information indicators are constructed by integrating various factors of tourism security. In the third part, the optimization algorithm of the tourism security early warning information system based on the LSTM model is trained and tested, and the simulation results are analyzed.

## 2. Related Work

The tourism security early warning information system contains a complex system of many influencing factors, which can evaluate and analyze various security indicators of tourism destination and determine the change trend of the system composed of the overall environment of tourism destination, so as to early warn and eliminate the security incidents that may occur in the security system [7, 8]. The tourism safety early warning information system can promote the sustainable development of tourism destination and improve the satisfaction of tourists' experience and personal safety and has important guiding significance in the long-term development of tourism industry and social economy, natural environment, and social stability [9]. Therefore, the research of the tourism security early warning information system has always been the focus of attention. Tourism safety factors are diversified, and their external manifestations can be roughly divided into natural disasters, diseases, crimes, traffic safety, and others. Many of them are uncontrollable, but scenic spots can still analyze some potential risk factors according to the analysis of relevant information. Some scholars have proposed an Intelligent Tourism early warning system for the stampede in scenic spots, that is, to analyze and guide the monitored data through intelligent services and processing functions [10]. This method is more suitable for use in urban scenic spots, and its early warning focuses on the tourism safety problems caused by human factors. According to the characteristics of natural scenic spots, some scholars proposed to establish the risk identification and evaluation model of natural scenic spots through the combination of the GIS and Bayesian network model [11]. This method has strong pertinence and can clarify the scope of risk and improve the accuracy of tourism safety early warning, but it needs long-term effective data as the basis of decision-making, which greatly increases the time cost. Some scholars proposed to build a safety early warning system based on the BP neural network. Its modeling is relatively simple and can obtain information analysis results in a relatively short time [12]. However, the BP neural network is weak in the analysis of time series information, and its output early warning results tend to static analysis. And with the increase of the types of risk factors, its accuracy is also affected to a certain extent. In addition, some research on tourism security early warning mostly focuses on the application mechanism of the artificial neural network in tourism security emergencies, which provides theoretical support and lays a solid theoretical foundation for tourism security research [13]. In addition, according to the current situation of tourism environment, researchers put forward to explore the ecological deterioration and sudden environmental security problems caused by tourism activities from an ecological perspective, predict the ecological environment status of tourism destinations, and make targeted preventive measures and rescue plans [14]. However, from the aspect of tourism security crisis early warning and management, the tourism security early warning system based on the BP neural network still has many deficiencies in processing time series data and needs to be further optimized.

The main objects of tourism security early warning system are tourists or local residents [15, 16]. Therefore, the information it provides is more detailed, which has a good effect in the security of outbound tourism. However, some travellers ignore early warning information or do not pay attention to relevant early warning information in time, and they do not pay attention to early warning information and suggestions [17]. It should be noted that the tourism safety early warning information system does not specifically establish a long-term safety early warning information system for tourism, but is issued by the relevant meteorological bureau, and the Safety Supervision Bureau and other departments carry out classified early warning for natural disasters and social security events, and the information subject is not limited to tourists [18, 19]. A similar tourism security early warning information system has been established, and the warning language is relatively mild. This paper briefly introduces the tourism destination countries, but it does not clearly classify the contents of early warning [20]. At the same time, citizenship does not connect tourism services, so few people pay attention to the released tourism security early warning information [21, 22]. Researchers have been constantly trying and studying, hoping to build a more scientific tourism security early warning information system [23].

### 2.1. Construction and Optimization of Tourism Security Early Warning Information System Based on LSTM

The tourism safety early warning information system is used to predict and warn the changes of scenic spots in the future from multiple dimensions according to the reasonable index system and scientific methods. Therefore, the influencing factors of tourism safety early warning information are diversified and nonlinear. In this paper, the LSTM model is used to construct the tourism safety early warning information system, which improves the processing ability of the system to temporal information, so as to realize the purpose of real-time dynamic information supervision and analysis.  Figure 1 shows the flowchart of the tourism security early warning information system based on the LSTM model.

### 2.2. Construction of Tourism Safety Early Warning Neural Network Information System

The artificial neural network which simulates the connection between human neurons can process the relevant signals, obtain the data signal prediction model, and solve the nonlinear data prediction and other related problems. Therefore, this paper selects the BP neural network as the foundation of the tourism security early warning information system and extracts the implicit relationship of the static data that need to be analyzed and predicted [24]. The neurons of the BP neural network can connect multiple inputs but only have one output node, as shown in Figure 2.

The input layer of the multilayer perceptron is represented as *L*_in_ and *x*=(*x*_1_, *x*_2_, *x*_3_)^*T*^, the hidden layer as *L*_hidden_ and *h*=(*h*_1_, *h*_2_, *h*_3_, *h*_4_)^*T*^, and the output layer as *L*_out_ and *y*=(*y*_1_, *y*_2_, *y*_3_). The process of data transmission from input layer to output layer is forward propagation, as shown in

(1) $$\begin{array}{c} h=f\left(W^{1T}x+b^{1}\right), \end{array}$$

(2) $$\begin{array}{c} y=f\left(W^{2T}x+b^{2}\right). \end{array}$$

The weight matrix of data transfer is expressed as *W*^1^ ∈ *R*^3×4^; the weight of data transfer connection between hidden layer and output layer is expressed as *W*^2^ ∈ *R*^4×3^, and the bias of output layer is expressed as *b*^2^ ∈ *R*^3×1^. The activation function *f* is shown in

(3) $$\begin{array}{c} f=\frac{1}{1+\exp\left(-x\right)}. \end{array}$$

In the learning process of the BP neural network, the weights and thresholds are modified by the gradient method. The iterative formulas after the rest are shown in

(4) $$\begin{array}{c} \left\{\begin{array}{c} \Delta W\left(n+1\right)=-\eta \frac{\partial E}{\partial W\left(n\right)}+a\cdot \Delta W\left(n\right),\\ \Delta \theta \left(n+1\right)=-\eta \frac{\partial E}{\partial \theta \left(n\right)}+a\cdot \Delta \theta \left(n\right), \end{array}\right. \end{array}$$

(5) $$\begin{array}{c} \left\{\begin{array}{c} \Delta W\left(n+1\right)=W\left(n+1\right)-W\left(n\right),\\ \Delta \theta \left(n+1\right)=\theta \left(n+1\right)-\theta \left(n\right). \end{array}\right. \end{array}$$

Although the BP neural network can solve the nonlinear problem, the data processed by the BP neural network have no correlation on the time line; that is, it cannot process the time series characteristic data related to the last moment or earlier data. An LSTM is designed based on the structure of the BP neural network. The structure of function of network memory, that is, it can effectively remember the data characteristics of time dimension in training data, and its structure is shown in Figure 3.

The difference between the LSTM and BP neural network is that the nodes between the hidden layers are interconnected, so that the input of the hidden layer at that time contains two parts, that is, the output transmitted by the input layer at this time and the output of the hidden layer at the last moment, so that the hidden layer contains the information memory at this time and at the last moment or earlier [25]. The transfer process is shown in

(6) $$\begin{array}{c} h_{t}=f\left(W^{1T}x_{t}+W^{hT}h_{t-1}+b^{1}\right), \end{array}$$

(7) $$\begin{array}{c} y_{t}=f\left(W^{2T}h_{t}+b^{2}\right). \end{array}$$

And *b*^2^ represents the output layer offset. When the time is *t*, the input is *x*_*t*_, the hidden layer output is *h*_*t*_, and the output is *y*_*t*_; when the time is *t* − 1, the hidden layer output is *h*_*t*−1_. The activation function formula is shown in

(8) $$\begin{array}{c} \tanh\;x=\frac{\sinh\;x}{\cosh\;x}=\frac{e^{x}-e^{-x}}{e^{x}+e^{-x}}. \end{array}$$

The sum of the losses is the total loss function. Let the loss function be labeled as the negative log likelihood function, as shown in

(9) $$\begin{array}{c} L^{t}=-y^{t}\log\;o^{t}. \end{array}$$

Then, the total loss function of the sequence is shown in

(10) $$\begin{array}{c} L\left(\left\{x^{1},\ldots ,x^{t}\right\},\left\{y^{1},\ldots ,y^{t}\right\}\right)=\sum L^{t}. \end{array}$$

The development of LSTM can be transformed into the corresponding BP neural network and trained by the BPTT algorithm [26, 27]. If it is necessary to train *t* time data, the LSTM is expanded into a BP neural network with *t* hidden layer. It can be seen from Figure 2 that the parameters in the same position after the expansion of the LSTM are shared with each other, while the BP neural network is not shared, so the LSTM greatly reduces the learning and training parameters. According to the relevant theory, it can be considered that the length of the sequence data that can be processed by LSTM is infinite, and the hidden layer of processing information is also infinite. Therefore, in the actual information transmission process, the information in the hidden layer neurons will gradually weaken and lose due to the extension of time, that is, the gradient vanishing phenomenon. This leads to the decrease of prediction performance. In addition, the length of the delay window needs to be determined in advance when the LSTM is trained, which improves the difficulty of automatically obtaining the optimal parameters in practical application.

### 2.3. Optimization of Tourism Security Early Warning Information System Based on LSTM

In order to solve the above problems of LSTM, so as to make its memory long-term, Figure 4 shows the LSTM structure development diagram.

It can be seen from the figure that the LSTM neural network introduces controllable, so as to avoid the gradient disappearance problem of LSTM. There are four layers in LSTM cell, including forgetting gate, input layer, output layer, and update layer, which interact with each other in a special way. And we provide corresponding continuous writing, reading, and reset functions. That is to say, the LSTM neural network adds a C state for long-term information memory on the basis of the recurrent neural network, which is the unit structure of LSTM. If the time at this time is *t*, when the forgetting gate layer controls the amount of information transferred from the previous unit state *c*_*t*−1_ to the current *c*_*t*_ state,

(11) $$\begin{array}{c} f_{t}=\sigma \left(w_{f}*\left[h_{t-1},x_{t-1}\right]+b_{f}\right). \end{array}$$

The main purpose of the input gate is to filter information to avoid useless information entering the current *c*_*t*_ state. The sigmoid layer and tanh layer of the input gate can update the state. The formulas are shown in

(12) $$\begin{array}{c} i_{t}=\sigma \left(w_{i}+\left[h_{t-1},x_{t}\right]+b_{i}\right), \end{array}$$

(13) $$\begin{array}{c} g_{t}=\tanh\left(w_{c}*\left[h_{t-1},x_{t}\right]+b_{c}\right), \end{array}$$

where *σ* is sigmoid function and the numerical range is [0, 1]. After that, the last moment state *c*_*t*−1_ and *f*_*t*_ are multiplied to update the state. The useless information is filtered out, and a new value *i*_*t*_*∗g*_*t*_ is added. The corresponding adjustment is made according to the individual update state. The formula is shown in

(14) $$\begin{array}{c} c_{t}=f_{t}*c_{t-1}+i_{t}*g_{t}. \end{array}$$

The output gate is used to control the current output affected by long-term storage information. It mainly determines the cell to be output through sigmoid layer, then sets the cell in [−1, 1] range by tanh, and multiplies the corresponding output gate. Finally, the determined output part is output, as shown in

(15) $$\begin{array}{c} o_{t}=\sigma \left(w_{0}*\left[h_{t-1},x_{t}\right]+b_{0}\right), \end{array}$$

(16) $$\begin{array}{c} h_{t}=o_{t}*\tanh\left(c_{t}\right). \end{array}$$

It can be seen from the above formula that sigmoid function is the activation function of input, output, and forgetting gates with values in [0, 1]. The other activation function, tanh, as shown in formula (6), is also commonly used in the input and output gates of LSTM, and its monotonicity is more consistent with the characteristics of neurons in neural networks.  Figure 5 shows two kinds of activation function diagrams.

### 2.4. Index Construction of Tourism Security Early Warning Information System

Tourism safety includes many influencing factors. According to the relevant analysis and induction, the index of tourism early warning information system in this paper is three levels, that is, the first level is tourism safety early warning, and the second level has four indicators, that is, the stability of tourism natural disasters, the safety of Tourism travel facilities, the safety of tourism destinations, and the safety of tourism environmental pollution. In addition, each first level indicator also contains three levels of impact factors.

Tourism safety early warning mode is divided into excellent level, good level, qualified level, and critical level. Among them, the excellent level indicates that the overall environment of the tourism destination has high security, there is no hidden danger, and there is no need to worry about the occurrence of emergencies. Good level means that the overall environment of the tourism destination has high security. Although there may be potential safety hazards and the possibility of small-scale security emergencies, the probability of occurrence is very small, and there are sound and mature treatment plans and remedial measures. From the perspective of realistic probability, potential tourism safety accidents may occur. However, the impact of such accidents can be effectively controlled within the corresponding range, and there is a good response plan, which requires tourists to have a certain degree of cognition and knowledge of potential safety hazards. Tourists who do not have this condition are not encouraged to enter the tourist destination. The critical level means that the tourism destination has a high probability of serious tourism safety accidents, and because there is no corresponding treatment plan and measures, once a safety accident occurs, it will have serious or even catastrophic consequences for tourists and the tourism destination. Tourists should be prevented from entering the tourism destination within this level. In order to show the four tourism safety early warning modes more intuitively, the four level alarms are matched with corresponding early warning signals, that is, the safety level early warning signal is green, the good level early warning signal is blue, the qualified level early warning signal is orange, and the critical level signal light is red.  Figure 6 shows the warning value and discrimination mode of tourism security early warning.

### 2.5. Test Results of Tourism Security Early Warning Information System Based on LSTM

#### 2.5.1. Optimization Test Results of Tourism Security Early Warning Information System Based on LSTM

In the LSTM algorithm, the time step represents the length of the index sequence that can be used, which has a certain impact on the model. Therefore, under the condition that the algorithm remains unchanged, the performance of the algorithm with the step size of 4, 45, and 90 is tested, as shown in Figure 7.

It can be seen from the results in the figure that the LSTM algorithm will continuously improve the corresponding prediction performance with the increase of time step. When the time step increases to a certain length, the accuracy of LSTM algorithm decreases. In addition, the time step can reflect the correlation length of the data in the time series. If the time step is too short, the correlation information between the data will be insufficient, which will reduce the prediction effect of the algorithm. When the step length is too long, it will reduce the correlation between the data because of too much redundant data, thus reducing the prediction accuracy of the algorithm, so the selection of the step length algorithm is very important.

According to the LSTM recurrent algorithm, the increase of the number of layers will improve the learning performance, but layers will also lead to the improvement of the complexity of the algorithm system, affect its convergence speed, consume more time in the sample training, and increase the difficulty of training. Therefore, this paper tests the performance of the LSTM algorithm, as shown in Figure 8.

In the figure that the convergence effect of LSTM improves with the increase of layers, but the corresponding training and testing time is also longer and longer. And when the number of layers of LSTM increases to four, the improvement of its performance is not obvious, but it takes a long time. Therefore, considering the needs of all aspects, the three-layer LSTM algorithm is the most appropriate. As shown in Figure 9, the hidden layer of LSTM algorithm contains different numbers of node loss function values.

It can be seen from the figure that when the number of hidden layer nodes reaches 520, the loss function value of the LSTM algorithm reaches the minimum. Compared with the loss function of the hidden layer with 130 and 260 nodes, it can be seen that with the increase of the number of nodes, the corresponding loss function value decreases significantly. This shows that when the number of hidden layer nodes is large enough, the fitting performance of the LSTM algorithm can be brought into full play.

### 2.6. Simulation Test Results of Tourism Security Early Warning Information System Based on LSTM

As shown in Figure 10, it is the error comparison chart of the BP neural network algorithm and LSTM algorithm for tourism safety index prediction results. In the results of the figure, the prediction result of the LSTM algorithm is closer to the real value. The algorithm has a large error in the prediction results of individual values, mainly because the BP neural network is prone to the problem of local optimal solution. Therefore, in terms of accuracy and stability, the prediction accuracy of LSTM for time series data is higher and the stability is better.

As shown in Figure 11, it is an early warning analysis model information system based on LSTM. Tourism destination security is a complex dynamic change, so the input value of the tourism security early warning information system can be not only discrete variables but also continuous variables, and the output value belongs to Boolean discrete vector.

The security status of tourism destination is divided into different levels, and the output value information system based on LSTM is set as a vector between 0 and 1. When the *m*-th index element represents 1 and the other index elements represent 0, the security of tourism destination is in a certain level. The simulation test results the tourism security early warning information system as shown in Table 1.

## 3. Conclusion

With the continuous development of economy, people begin to see the difference of the world through tourism on the basis of meeting the basic life. However, what is not matched with the booming tourism industry is the tourism security early warning information system. Tourism security is a comprehensive problem composed of many factors, which is not only related to the life and property safety of tourists, but also related to social stability, and the development and protection of tourism resources. At present, the tourism is relatively backward, focusing on the remedial measures and treatment after the occurrence of security incidents, which cannot play the role of early warning to reduce disaster losses. Therefore, this paper studies the optimization algorithm of the tourism security early warning information system based on LSTM. On the basis of the tourism security based on the BP neural network, it uses recurrent neural network and LSTM to optimize the system algorithm, so as to improve the ability of the early warning information system to process and predict the time series data. The experimental results show that the learning ability and convergence effect of LSTM model will improve with the increase of the number of hidden layers, but when it increases to a certain number, the increase of learning ability and convergence effect is not obvious. Therefore, it is necessary to set an appropriate number of hidden layers for the LSTM model to improve its performance. The tourism security early warning information system based on the LSTM model has better accuracy and stability than the tourism security early warning information system based on the BP neural network algorithm, has better processing and prediction ability for time series data, and is more in line with the needs of the tourism security early warning information system. In addition, compared with other methods, the tourism security early warning information system based on the LSTM model can be applied to a wider range, whether it is a tourist city scenic spot or a tourist natural scenic spot, or it can be combined with intelligent wearable devices for data collection and analysis. However, the experimental data in this paper are mainly for the analysis of the indicators of the scenic spot, so the index system needs to be further improved. In the future development, the tourism safety early warning information system between scenic spots should be connected with each other to strengthen the information circulation. At the same time, set up a tourism safety early warning information subsystem for economically underdeveloped scenic spots to reduce the cost of tourism safety early warning information system on the basis of ensuring the safety of scenic spots and tourists.

## Figures and Tables

**Figure 1:** Flowchart of the tourism security early warning information system based on the LSTM model.

**Figure 2:** BP neural network simple model.

**Figure 3:** The structure of network memory function.

**Figure 4:** LSTM structure expansion.

**Figure 5:** Two activation function diagrams.

**Figure 6:** Warning value and discriminant model of tourism safety.

**Figure 7:** LSTM recursive neural network algorithm does not synchronize the long performance test.

**Figure 8:** LSTM recursive neural network algorithm was used to test the level dependent performance.

**Figure 9:** The hidden layer of the LSTM recursive neural network algorithm contains different numbers of node loss function values.

**Figure 10:** The error comparison graph of the BP neural network algorithm and LSTM recursive neural network algorithm for tourism safety index prediction results.

**Figure 11:** An early warning analysis model of the tourism security early warning information system based on the LSTM recursive neural network.

**Table 1:** Based on LSTM recursive neural network tourism security early warning information system simulation test results.

	X1	X2	X3	X4	X5	X6	X7	X8	X9	X10	Alarm indication
1	0.95	0.74	0.089	0.06	0.02	0.72	0.44	0.04	0.03	0.12	(1000) green
2	0.87	0.61	0.06	0.11	0.05	0.67	0.36	0.15	0.06	0.11	(1000) green
3	0.74	0.66	0.14	0.16	0.08	0.67	0.44	0.20	0.09	0.16	(0100) blue
4	0.67	0.51	0.16	0.17	0.07	0.54	0.34	0.28	0.12	0.32	(0010) orange
5	0.82	0.67	0.08	0.11	0.05	0.68	0.39	0.15	0.06	0.14	(0100) blue
6	0.58	0.58	0.16	0.20	0.09	0.50	0.27	0.31	0.15	0.22	(0010) orange
7	0.62	0.48	0.27	0.20	0.12	0.50	0.25	0.36	0.22	0.32	(0001) red
8	0.57	0.41	0.21	0.22	0.15	0.42	0.28	0.44	0.27	0.51	(0001) red

## Data Availability

The data used to support the findings of this study are available from the corresponding author upon request.
